The article "Network Extraction and Analysis of Character Relationships in Chinese Literary Works" was published in 2022. Journal: Comput Intell Neurosci.

# Network Extraction and Analysis of Character Relationships in Chinese Literary Works

**DOI:** 10.1155/2022/7295834

**Published:** 2022-05-14

**Authors:** Chao Fan, Yu Li

**Affiliations:** ^1^The School of Artificial Intelligence and Computer Science, Jiangnan University, Wuxi 214122, China; ^2^Jiangsu Key Laboratory of Media Design and Software Technology, Jiangnan University, Wuxi 214122, China

## Abstract

Character relationships in literary works can be interpreted and analyzed from the perspective of social networks. Analysis of intricate character relationships helps to better understand the internal logic of plot development and explore the significance of a literary work. This paper attempts to extract social networks from Chinese literary works based on co-word analysis. In order to analyze character relationships, both social network analysis and cluster analysis are carried out. Network analysis is performed by calculating degree distribution, clustering coefficient, shortest path length, centrality, etc. Cluster analysis is used for partitioning characters into groups. In addition, an improved visualization method of hierarchical clustering is proposed, which can clearly exhibit character relationships within clusters and the hierarchical structure of clusters. Finally, experimental results demonstrate that the proposed method succeeds in establishing a comprehensive framework for extracting networks and analyzing character relationships in Chinese literary works.

## 1. Introduction

Classic literary works are passed down to the present day because imaginative virtual worlds created by the authors can reflect many characteristics of our society. Character relationships in a novel indirectly reflect the writer's experiences and feelings about social life, cultural beliefs, and habits. Traditional analysis tries to discover the value of a literary work and compares similarity between the social structure in the work and real-world structure. However, recent analysis paid more attention to social relationships of characters. For example, the relationships of characters portrayed by a novel often carry a large amount of social information which is important for scholars when interpreting a literary work. Hence, extracting a social network and analyzing intricate character relationships will help to better understand the internal logic of plot development and explore the significance of a literary work. For instance, it can ease the process of reading a novel with too many characters, because readers are often confused about complicated character relationships while reading a long novel.

This paper attempts to extract networks of character relationships for several Chinese literary works by performing network analysis, cluster analysis, and data visualization. By applying these technologies and refining shared features in literary works, we succeeded in building a framework for studying network extraction and character relationship analysis of the Chinese literature. Initially, a Chinese lexical analysis on the novel text is used to resolve character names. Co-word network analysis is then employed to extract a network of character relationships. By analyzing the created network, we are able to grasp the basic characteristics of important characters in the specified Chinese novel. Finally, a variety of data visualization techniques are proposed to display character relationships in the novel.

This article is arranged as follows: Related researches are discussed in Section 2.  Section 3 elaborates the methodology of character relationship extraction and analysis in Chinese literary works. Datasets and experimental results are described in detail in Section 4. The conclusion is drawn in Section 5.

## 2. Related Work

Analyzing literary works quantitatively by using scientific tools is one of the current research hotspots. The research approach is mainly divided into three categories: language analysis, text analysis, and comprehensive analysis [1]. Experts in both literature and computer science have recently focused on comprehensive analysis, which will be the main direction for literary research in the future. Zhao et al. [2] established a model of character graphs based on emotional polarity and gave general procedures to comprehend the Chinese literature. Huang et al. [3] developed a Chinese person entity relation extraction technology utilizing distant supervision, which can automatically identify and extract semantic relationships. Li and Liu [4] divided the corpus of a classical Chinese novel into training data and test data. Based on an N-gram language model and a random forest algorithm, they extracted features and performed a classification experiment to identify the authorship of the novel.

Social networks have also been introduced to analyze literary works. A growing number of scholars have begun to research literary character relationships based on social networks. Muhuri et al. [5] devised a means of annotation and character categorization to extract social networks. They applied it to two Bengali dramas and successfully found the protagonist and antagonist in the literature. Chowdhury et al. [6] investigated character relationships in a novel and its adapted film based on social network. They exploited many network features such as centrality metrics to analyze the difference in the character categorization within two expressions of art. Wang et al. [7] utilized co-word and social network analyses to study old Chinese literature in the Qing Dynasty. Fan et al. [8] examined character relationships in a classical Chinese novel by combining social network and cluster analysis.

A scheme for constructing a social network is using the co-word analysis technique. It measures the strength of relationships by counting the co-occurrence of words in a text. In recent years, co-word analysis has been widely employed in several fields. Chen et al. [9] conducted research by collecting the scientific literature with the topic of medical image processing. In order to explore research hotspots in this field, keywords of papers were used for co-word and cluster analysis. Huang et al. [10] chose industrial symbiosis as their research topic, using co-word and social network analysis to evaluate the current status and trends. They found that this research direction showed an interdisciplinary characteristic. Another research [11] built and visualized a co-word network in the Night-Time Light remote sensing field according to data from the Web of Science. Hu et al. [12] adopted scientometrics and co-word analysis to study bibliographic data in food safety from 1991 to 2018. Their work focused on food safety in agriculture and industry and revealed global research trends in this field. Xie et al. [13] predicted the evolution of academic research and hotspots in bioacoustics and ecoacoustics based on bibliometric analysis and network-based methods such as co-word network analysis, co-author network analysis, and co-citation network analysis.

## 3. Methodology

Manual analysis is a choice when the number of characters is small in a literary work. Nevertheless, it is unacceptable to manually process a novel with hundreds and thousands of characters. Thus, this paper focuses on automatically extracting and analyzing character relationships with the help of social networks and natural language processing technologies. The main framework of character relationship analysis can be illustrated in Figure 1. At first, a corpus of the Chinese literature and its corresponding character name list are loaded. Chinese lexical analysis is then performed so that character names can be correctly resolved. After building a social network based on co-word analysis, we calculate the number of network features and implement the visualization of network data in many ways.

### 3.1. Preprocessing

Before preprocessing, a full-text collection of Chinese literary works has to be collected from open datasets on the Internet. A selected literary work should contain the standardized Chinese text with high quality. Besides, a corresponding character name list downloaded from the web has to be provided for co-word analysis. Data cleansing is also done to correct some mistakes and remove unclear data in a raw corpus.

A Chinese natural language processing tool, ICTCLAS (https://ictclas.nlpir.org/), was used to perform lexical analysis, including segmentation, part-of-speech (POS) tagging, and named entity recognition (NER). Combining the character name list and character names resolved by NER, we succeeded in preparing the data for constructing a character relationship network.

### 3.2. Network Extraction of Character Relationships

Literary character relationships can be described as an undirected network. The character name is recognized as the node, and co-appearance of two names in a sentence or a paragraph is deemed as the link. Then, the weight of a link can be calculated by counting the number of times that the two names co-occur in the text. By performing co-word analysis, we can extract a weighted network of character relationships for the Chinese literature.

When dealing with Chinese character names, it is necessary to identify a character with different types of names: full name, nickname, and abbreviated name. A powerful algorithm should handle it correctly and effectively. We set a series of rules to convert names of different forms into full names.

### 3.3. Network Analysis for Character Relationships

Performing network analysis requires calculating multiple network features. The network features involve degree distribution, density, clustering coefficient, average clustering coefficient, shortest path length, average shortest path length, diameter, and centrality.

The degree of a node represents the number of its neighbors in the network. Degree distribution [14] is defined as the distribution of node degree, showing how links are distributed among nodes. Many researchers inspect whether a character relationship network has the power-law distribution, which is a common pattern discovered in numerous real networks [15].

Network density assesses the relative denseness of a network from the perspective of connected links. In a network, density is the portion of potential links which actually exist in the network [8]. It is often used in social networks to measure the intensity of social relationships and trends in evolution.

As a local feature of a network, the clustering coefficient [16] reflects the degree of clustering from the perspective of the nodes. It is the number of existing connections within a node's neighbors divided by the number of potential connections [17]. If all neighbors of a node are connected to each other, the clustering coefficient of this node will be 1. The average clustering coefficient, also known as the clustering coefficient of a network, is an average of all nodes' clustering coefficients. This value indicates the probability that friends of a person are also friends in real social connections.

The shortest path length [18] between two nodes refers to the number of links that connects two nodes by the shortest path. Thus, the average shortest path length is defined by the average number of links along the shortest paths. It measures information transmission efficiency within a network. Another indicator related to the shortest path is the diameter of a network, which is the maximum value of all shortest path lengths.

Centrality [15] is a measurement of significance for each node in the network. Three centralities are often discussed in network science involving degree centrality, betweenness centrality [19], and closeness centrality [20]. They are calculated based on the concept of degree, betweenness, and degree of closeness.

### 3.4. Cluster Analysis for Character Relationships

The weight of a link between two nodes in a social network can be used to represent the similarity of two characters. The larger the weight is, the more likely the two characters will be related to each other. At the beginning, a co-occurrence matrix is created by counting the weights of links, which are frequencies of character names appearing together. Furthermore, Ochiai coefficients [21] are calculated to implement the normalization of the co-occurrence matrix for the purpose of eliminating the influence of frequency of a character existing in a literary work. The formula of the Ochiai coefficient is described by

(1) $$\begin{array}{c} \text{Och}=\frac{\text{freq}\left(X\cap Y\right)}{\sqrt{\text{freq}\left(X\right)\times \text{freq}\left(Y\right)}}, \end{array}$$

where freq(*X*) is the frequency of character *X* and freq(*X*∩*Y*) is the frequency that *X* and *Y* co-occur in the literary work. In addition, a similarity matrix can be produced by applying the mathematical formula to the co-occurrence matrix. The elements of the similarity matrix range from 0 to 1. A large value implies a high similarity between the two characters, which means they incline to gather together in cluster analysis.

After taking the similarity matrix of character relationships as input, we exploit a bottom-up agglomerative hierarchical clustering method to organize characters into groups. The algorithm treats each character as a cluster at first. Two most similar clusters are merged at each iteration until only one cluster remains or it reaches the specified threshold. Finally, a hierarchical tree structure of character relationships is obtained through cluster analysis.

### 3.5. Data Visualization

Data visualization offers a graphical representation of data, helping us better understand the pattern within the data. Character relationships can be visualized in many different types. In this paper, clustering results of characters are portrayed in the form of a dendrogram. Since the output of hierarchical clustering is a binary tree, a tree-like dendrogram is an effective structure for visualizing character relationships.

Furthermore, the binary tree can be illustrated by a Venn diagram [22] as shown in Figure 2. In Figure 2, a red leaf node is also a node in the Venn diagram. The red node represents a character in the literary work, whereas a branch node stands for a larger group involving characters or small groups. Using the Venn diagram to display the result of hierarchical clustering has the following advantages: for one thing, nodes can be connected by links in the Venn diagram, which cannot be done in a tree structure; for another, the Venn diagram can clearly express a hierarchical structure. According to Figure 2(b), cluster A contains cluster B and character C, whereas characters D and E are included in cluster B.

However, application of a simple Venn diagram has some limitations. For instance, a novel with *n* characters incorporates *n* − 1 clusters in the hierarchical clustering result. When the number of characters is too large, there will be a plethora of nodes and groups in the Venn diagram. It leads to a poor visualization of clustering results. There is no need to depict all clusters in the hierarchical structure, because researchers only pay attention to several important clusters. This paper improves the representation of target clusters by removing internal small clusters and retaining all character nodes. As shown in Figure 3, inner cluster B will be omitted if we are interested in cluster A, which results in a simplified visualization. The simplification of the Venn diagram is very useful when we visualize a multitude of characters with a small number of clusters.

## 4. Experimental Results

### 4.1. Datasets of Chinese Literary Works

A myriad of e-books of the Chinese literature can be downloaded from the Internet. In this paper, four classical Chinese novels are chosen as datasets to be analyzed. The novels' names and their abbreviations are presented in Table 1. Original texts are preprocessed to meet the experimental criteria. Cleaned data are available from the authors upon request. As character names are indispensable to extract social network from a literary work, character name lists of novels are also collected through the Internet. The number of characters for each novel is given in Table 1.

### 4.2. Results of Network Extraction and Analysis

Based on the character name list and co-word analysis, a social network of character relationships is extracted for each Chinese novel. Taking Demi-Gods and Semi-Devils (DGSD) as an illustration, a network with 169 nodes and 1,559 links is established in this paper. Figure 4 gives the visualization of the DGSD network by showing the top-50 nodes in degree distribution. It is a weighted undirected network where the size of a node denotes the frequency of a character name appearing in DGSD and the strength of a link represents the co-occurrence of two names in different semantic contexts.

The degree distribution of four networks and their log-log plots are depicted in Figures 5 and 6, respectively. According to the figures, only the degree distribution of the RTK network follows a power-law distribution—a significant property of the real-world network. In the log-log plot of Figure 6, we can fit a linear equation to the data of RTK well. However, other datasets of literary works fail to capture power-law properties because their authors only write a small number of core characters and neglect most low-frequency characters.

The average degree of a character relationship network means how many neighbors does a character connect on average. The indices for the 4 Chinese novels are listed in Table 2. The DRM network has the largest average degree. It means that characters in DRM are closely joined together in comparison with other novels. On the contrary, the RTK network has the smallest average degree because its author describes a large number of characters who appear only once or twice in the novel.

According to Table 2, densities of the four networks are less than 0.3, so they are sparsely connected networks, especially the RTK network. The average shortest path length is more than 3 for the RTK network but less than 2 for the DRM and LCH networks. Distribution of the shortest path length between two nodes is displayed in Figure 7. As for diameter which represents the distance of the largest-shortest path, only the RTK network has a diameter of 9, which is much larger than 4. Therefore, it has to afford a high cost of reaching another node in the RTK network in comparison with the other three networks.

The clustering coefficient reflects the local characteristics of a node. In a Chinese literary work, a character with the largest clustering coefficient does not necessarily have the most important role. The average clustering coefficients for 4 novels are given in Table 2. Moreover, we compare the character relationship network with a randomized version of a network with the same number of nodes and links, obtainable with a configuration model [23] that keeps the same degree distributions. This type of a random model is better than a simple ER model [24, 25]. From the results obtained in Table 3, the average shortest path length of each character relationship network is smaller than that of a random network except for the RTK network. The exception may be originated from an apparent three-group structure existing in the RTK network. All character relationship networks have larger average clustering coefficients. Hence, the social network of character relationships in a literary work is often a small-world network.

Three centralities can be calculated to measure significance of characters in a novel. Degree centrality is proportional to the degree of a node, which highlights the pivotal position of a node. Betweenness centrality reflects the “communication” ability of a node in the network. A high-betweenness node has a stronger ability to communicate with others. Closeness centrality represents the degree of accessibility from one node to other nodes in the network. Taking the example of DGSD, the top ten characters in centrality are shown in Table 4. Eight of the ten characters appear in three rankings, incorporating Duan Yu, Xu Zhu, Heshang, Murong Fu, Wang Yuyan, Qiao Feng, A Zhu, and A Zi.

### 4.3. Results of Cluster Analysis and Visualization

In order to discover clusters from data, the co-occurrence matrix should be first created by counting the weights of links. An example of five characters in DGSD is presented in Table 5. The diagonal number is the frequency of a character's name appearing in the novel.

Normalization of the above co-occurrence matrix is finished by computing the Ochiai coefficient. Then, the co-occurrence matrix is converted into a similarity matrix as shown in Table 6.

Similarity of any two characters can be used for cluster analysis. In this research, a bottom-up hierarchical algorithm employing the similarity matrix is implemented to cluster character names in the literary work. As the result of hierarchical clustering is a binary tree, a dendrogram is drawn to describe character relationships in the novel.  Figure 8 depicts a dendrogram of the clustering result for 33 main characters in DRM. Four large clusters can be identified by the clustering algorithm, including the Jia family of the Rongguo Mansion (H1), the Jia family of the Ningguo Mansion (H2), the Xue family (H3), and a group of noble people (H4). In our algorithm, H1 and H2 are clustered together in the hierarchy, which is called the “Jia family.” Furthermore, the Jia family (H1 and H2) and the Xue family (H3) are combined to form a bigger cluster due to marriage. H4 is a group of noble people with titles that are closely connected. Finally, all the clusters are aggregated into one cluster.

Besides the dendrogram, an improved Venn diagram is also proposed to depict the hierarchical clustering result.  Figure 9 gives an instance of LCH using an improved method and reveals a visualization result by setting the number of clustering as 5. In this figure, small groups within 5 clusters are eliminated so that clusters can be clearly presented. Also, the hierarchical structure of 5 clusters is exhibited by filling different clusters with different colors. Moreover, we can control the number of clusters and merge nodes with the same cluster label in hierarchical clustering. The proposed visualization method can not only draw connections between nodes but also show the hierarchical structure of clusters. For example, four groups on the left side of Figure 9 are different gangs in mainland China. They cluster together to form a large group with leading Chinese characters. The group on the right side of Figure 9 is composed of Mongolian characters. Five groups are aggregated to build a small world of LCH with a hierarchical framework.

## 5. Conclusions

This article focuses on network extraction and analysis of character relationships in Chinese literary works. Four classical Chinese novels are selected as datasets to be analyzed. Initially, semantic segmentation and POS tagging were completed to process the raw corpus. A co-word analysis was then used to extract social networks of character relationships from Chinese literary works. Furthermore, a network analysis was performed by calculating degree distributions, network density, average clustering coefficient, centrality, and so forth. In order to implement cluster analysis, a co-occurrence matrix and similarity matrix were calculated to measure the similarity (or distance) between two characters in the network. Besides, data visualization was applied to explore character relationships. On the one hand, a tree-like dendrogram was used to display the result of hierarchical clustering. On the other hand, an improved Venn diagram was proposed to simplify graphical visualization. Finally, a dendrogram for DRM and a Venn diagram for LCH were visualized in our experiments.

In future, pronouns will be translated into character names using the coreference resolution so as to improve the extraction effect of character relationships. Introducing other network features and visualization approaches is another direction in the following research.

## Figures and Tables

**Figure 1:** Research framework for analyzing character relationships in Chinese literature.

**Figure 2:** Visualization of the outcome of hierarchical clustering. (a) A binary tree. (b) A Venn diagram.

**Figure 3:** Removal of internal clusters in the Venn diagram.

**Figure 4:** A visualization of the DGSD network with the top-50 nodes in degree distribution.

**Figure 5:** Degree distribution of the character relationship network. (a) DRM. (b) RTK. (c) LCH. (d) DGSD.

**Figure 6:** Log-log plot of degree distribution. (a) DRM. (b) RTK. (c) LCH. (d) DGSD.

**Figure 7:** Distribution of the shortest path length. (a) DRM. (b) RTK. (c) LCH. (d) DGSD.

**Figure 8:** Dendrogram of clustering result for the DRM network.

**Figure 9:** Improved Venn diagram visualizing the clustering result of LCH.

**Table 1:** Four Chinese novels selected as datasets.

Number	Chinese novel name	Abbreviation	Number of characters
1	Dream of the Red Chamber	DRM	265
2	Romance of the Three Kingdoms	RTK	1,133
3	Legend of the Condor Heroes	LCH	90
4	Demi-Gods and Semi-Devils	DGSD	169

**Table 2:** Basic network features of character relationship networks.

Network features	DRM network	RTK network	LCH network	DGSD network
Number of nodes	265	1,133	90	169
Number of links	4,748	5,844	1,013	1,559
Density	0.1357	0.0091	0.2529	0.1098
Average degree	35.83	10.31	22.51	18.45
Average shortest path length	1.9512	3.1743	1.7958	2.0889
Average clustering coefficient	0.7209	0.5306	0.7262	0.5907
Diameter	4	9	4	4

**Table 3:** Comparison with random networks generated by using configuration models.

Network	Type	Number of nodes	Number of links	Average shortest path length	Average clustering coefficient
DRM	Original	265	4,748	1.9512	0.7209
	Random			2.0345	0.3349

RTK	Original	1,133	5,844	3.1743	0.5306
	Random			3.0212	0.0824

LCH	Original	90	1,013	1.7958	0.7262
	Random			1.9034	0.3308

DGSD	Original	169	1,559	2.0889	0.5907
	Random			2.1423	0.2690

**Table 4:** Top ten characters of DGSD in centrality.

Ranking	Degree centrality	Betweenness centrality	Closeness centrality
1	Duan Yu (0.5952)	Duan Yu (0.1599)	Duan Yu (0.6696)
2	Xu Zhu (0.4405)	Xu Zhu (0.0833)	Xu Zhu (0.5874)
3	Heshang (0.4048)	Qiao Feng (0.0710)	Wang Yuyan (0.5675)
4	Murong Fu (0.3988)	Wang Yuyan (0.0508)	Heshang (0.5675)
5	Wang Yuyan (0.3929)	Heshang (0.0436)	Murong Fu (0.5627)
6	Qiao Feng (0.3690)	A Zi (0.0370)	A Zhu (0.5534)
7	A Zhu (0.3690)	Murong Fu (0.0332)	Qiao Feng (0.5511)
8	Duan Zhengchun (0.3333)	A Zhu (0.0323)	Duan Zhengchun (0.5379)
9	Duan Yanqing (0.3095)	Yelv Hongji (0.0244)	A Zi (0.5315)
10	A Zi (0.3036)	Bao Butong (0.0204)	Duan Yanqing (0.5315)

**Table 5:** An example of the co-occurrence matrix for DGSD.

Co-occurrence	Qiao Feng	Xu Zhu	Duan Yu	Xu Zhanglao	Xi Zhanglao	Jiumozhi
Qiao Feng	104	2	41	50	8	3
Xu Zhu	2	162	116	1	0	43
Duan Yu	41	116	286	1	1	127
Xu Zhanglao	50	1	1	53	1	0
Xi Zhanglao	8	0	1	1	10	0
Jiumozhi	3	43	127	0	0	173

**Table 6:** An example of the similarity matrix for DGSD.

Co-occurrence	Qiao Feng	Xu Zhu	Duan Yu	Xu Zhanglao	Xi Zhanglao	Jiumozhi
Qiao Feng	1	0.015408	0.23773	0.673466	0.248069	0.022366
Xu Zhu	0.015408	1	0.538912	0.010792	0	0.256855
Duan Yu	0.23773	0.538912	1	0.008122	0.018699	0.570949
Xu Zhanglao	0.673466	0.010792	0.008122	1	0.043437	0
Xi Zhanglao	0.248069	0	0.018699	0.043437	1	0
Jiumozhi	0.022366	0.256855	0.570949	0	0	1

## Data Availability

The original dataset used in this paper is available from the corresponding author on request.
